The article "Boosting Breast Cancer Detection Using Convolutional Neural Network" was published in 2021. Journal: J Healthc Eng.

# Boosting Breast Cancer Detection Using Convolutional Neural Network

**DOI:** 10.1155/2021/5528622

**Published:** 2021-04-03

**Authors:** Saad Awadh Alanazi, M. M. Kamruzzaman, Md Nazirul Islam Sarker, Madallah Alruwaili, Yousef Alhwaiti, Nasser Alshammari, Muhammad Hameed Siddiqi

**Affiliations:** ^1^Department of Computer Science, College of Computer and Information Sciences, Jouf University, Sakakah, Saudi Arabia; ^2^School of Political Science and Public Administration, Neijiang Normal University, Neijiang, China; ^3^Department of Computer Engineering and Networks, College of Computer and Information Sciences, Jouf University, Sakakah, Saudi Arabia

## Abstract

Breast cancer forms in breast cells and is considered as a very common type of cancer in women. Breast cancer is also a very life-threatening disease of women after lung cancer. A convolutional neural network (CNN) method is proposed in this study to boost the automatic identification of breast cancer by analyzing hostile ductal carcinoma tissue zones in whole-slide images (WSIs). The paper investigates the proposed system that uses various convolutional neural network (CNN) architectures to automatically detect breast cancer, comparing the results with those from machine learning (ML) algorithms. All architectures were guided by a big dataset of about 275,000, 50 × 50-pixel RGB image patches. Validation tests were done for quantitative results using the performance measures for every methodology. The proposed system is found to be successful, achieving results with 87% accuracy, which could reduce human mistakes in the diagnosis process. Moreover, our proposed system achieves accuracy higher than the 78% accuracy of machine learning (ML) algorithms. The proposed system therefore improves accuracy by 9% above results from machine learning (ML) algorithms.

## 1. Introduction

Breast cancer forms in breast cells and is considered as a very common type of cancer in women. Breast cancer is also a very life-threating disease of women after lung cancer. Breast cancer is categorized into various types according to the cell's appearance through a microscope. The two main types of breast cancer are (1) invasive ductal carcinoma (IDC) and (2) ductal carcinoma in situ (DCIS), with the latter evolving slowly and, generally, not having negative effects on the daily lives of patients. A low percentage of all cases (between 20% and 53%) are classified as the DCIS type; on the other hand, the IDC type is more dangerous, surrounding the entire breast tissue. Most breast cancer patients, approximately 80%, are in this category [1].

Breast cancer can be effectively treated through its early detection. Thus, the availability of proper screening methods is important for detecting the initial symptom of breast cancer. Various imaging techniques are used for the screening to identify this disease; the popular approaches are mammography, ultrasound, and thermography. One of the most significant methods of early detection for breast cancer is mammography. Ultrasound or diagnostic sonography methods are popularly used as mammography is not effective for solid breasts. Considering these issues, small masses can be bypassed by radiations from radiography and thermography may be more effective than the ultrasound technique in diagnosing smaller cancerous masses [2].

Due to the intrinsic difficulties associated with an image, with meagre contrast, noise, and lack of appreciation by the eye, instruments have been prepared to make and improve image processing. Nowadays, artificial intelligence (AI), machine learning (ML), and convolutional neural network (CNN) are the quickest rising areas of healthcare industry [1, 3–6]. AI and ML are found in the research arena that deals with and improves technological systems to resolve complex tasks through reducing necessity of human intelligence [7–9].

Deep learning (DL) which is part of machine learning family depended on artificial neural networks. DL architectures, such as DNN (deep neural networks), RNN (recurrent neural networks), DBN (deep belief networks), and CNN, are generally applied to the areas like computer vision, audio recognition, speech recognition, social network filtering, natural language processing, machine translation, drug design, bioinformatics, medical image analysis, materials scrutiny, histopathological diagnosis, and board game programs [10–12]. These new technologies, in particular DL algorithms, can be applied to improve the diagnostic accuracy and efficiency of cancer detection [13].

On the other hand, digital pathology (DP) is a way of digitalization of histology slides for producing high-resolution images. These digitized images are used for detection, segmentation, and classification through the application of image analysis techniques. Extra steps are required in deep learning (DL) using CNNs, such as digital staining, to understand patterns for image classification [14].

The opportunity that CNN brings to research on medical imaging is not restricted to deep CNN for extraction of the imaging feature. Indeed, a second field that can support medical research is the use of CNN for synthetic image rendering. Wahab and Khan [15] conducted a study by using MF-CNN (multifaceted fused-CNN) and a hybrid descriptor and revealed that, to assist with mitotic count-based selection of ROIs at lower resolution, acceptable color and textural characteristics are established. The MF-CNN recognizes several facets of the input picture to acknowledge dynamic patterns. It includes mitoses, excerpts, and handmade features from ROIs and uses the global image texture to shape a hybrid descriptor to train a classifier assigning WSIs scores. CNNs are opening up to unimaginable scenarios in areas where it is tedious for domain experts to develop successful features. Gravina et al. [16] noted that the naive use of CNNs might not be successful, since “medical images are more exceptional than normal images.” Mammographic lesion segmentation has been shown to be an effective source of knowledge, as it may help both extract shape-related structures and provide exact lesion localization.

An experiment was performed by Tsochatzidis et al. [17] to test the diagnosis of breast cancer with mammograms using CNN. They show that performance assessment in diagnosis is carried out on two datasets of mammographic mass such as DDSM-400 and CBIS-DDSM, with variations in the accuracy of the corresponding segmentation maps of ground truth. A computer-aided diagnosis (CAD) system was applied by Malathi et al. [18] for mammograms to allow initial identification, examination, and treatment of breast cancer. They discussed exploring a breast CAD architecture focused on characteristic fusion through deep learning of the CNN. The result reveals that the RFA (random forest algorithm) has the highest precision with less error than the CNN classifier (95.65 percent). The abnormality of the representations of the breast is investigated via the deep belief network (DBN). To discern the abnormal picture, the given work practices activate the contour segmentation and it may be ordered by the DBN. Desai and Shah [19] mentioned that deep comparison of the operation and architecture of each network is carried out and examination is then conducted based on the precision of the network's diagnosis and categorization of breast malignancy to assess which network outperforms the other. For the diagnosis and identification of breast cancer, CNN is observed to provide somewhat higher precision than MLP.

In prior research, Wahab and Khan [15] used CNNs to investigate the automated detection of IDC-type breast cancer. Several scholars used ML-based automatic detection techniques to detect the same. This aimed to obtain correct results to lessen the errors found in the diagnosis procedure. The study of Abdelhafiz et al. [20] also discovered that augmentation approach was fruitful in the automatic identification of this cancer, when using the given dataset. Another researcher [21] applied deep max pooling CNNs to identify images of mitosis in breast histology. The networks were competent to order the images based on pixel. A DL approach was used by Murtaza et al. [22] for the automatic identification and investigation of IDC tissue zones. Context-aware stacked CNNs were presented by Hossain [4] for the categorization of breast WSIs into simple, DCIS (ductal carcinoma in situ), and IDC (invasive ductal carcinoma). The system realized an area beneath the curve of 0.962 for the categorization of malignant and nonmalignant slides and obtained a three-class accurateness of 81.3% for WSI classification, demonstrating its potential for routine diagnostics. The works of Alhamid et al. [23] and Qian et al. [24] also presented some techniques to identify them. Their experiment results showed that the shearlet coefficients' magnitude and phase could enhance detection accuracy and generalizability.

Several previous studies have proposed using AI as well as CNN for image detection and healthcare monitoring [1, 18, 20, 25, 29]. But, for a medical side solution, which is around 60 percent for all class detection, 75 percent for only mass class, and 100 percent for only calcification, the accuracy percentage is too poor [26]. With the exception of only calcification argument, the accuracy of all argument and mass only argument can be further enhanced to obtain a better result [27]. Therefore, this research aims to increase precision level of breast cancer diagnosis using CNN. The current study proposes a system of breast cancer detection using several regression and DL techniques. The proposed system investigates several CNN architectures for the automatic detection of this type cancer. The proposed system initially uses a basic CNN and then adds it to three various architectures, all of which were guided by a big dataset of about 275,000, 50 × 50-pixel RGB image patches. The quantitative findings will be measured by validation tests. The two main objectives of this current research are, firstly, to present an automated tool for detecting IDC to lessen human mistakes in the process of diagnosis and, secondly, to examine the consequence of different types of CNN architecture in the proposed system. The remainder of this paper is organized as follows: The second section deals with materials and methods, the third section describes the results and discussions, and the final section deals with conclusion including recommendation, limitations, and future research.

## 2. Materials and Methods

### 2.1. Dataset

The dataset, Kaggle 162 H&E, was used for the proposed system [28]. Kaggle 162 H&E was also used by many researchers for similar kind of study [26, 30]. The data set consists of both benign and malignant images. Careful observation was ensured during splitting; the dataset was divided into validation data and testing data belonging to same distribution to well represent the model's generalized results. For learning indicators like weights and biases, training data is important, while validating data is essential for model verification and how exactly the model simplifies, thus tuning hyperparameters like learning rate and decay to boost the result of the model. A model's final output comes from precise work on the test results. To hold each pixel in the same range and prevent bias, the normalization has to be done on the whole image. Around 277,524 50 × 50-pixel RGB digital image patches were extracted from 162 WSI mounts scanned samples. All patches were labelled as 1 (IDC positive) or 0 (IDC negative).  Figure 1 presents examples of positive and negative tissues.

### 2.2. Data Process

All the patches are in RGB pixel format and are scaled from 0 to 255. We intended to apply machine learning (ML) classification methods to these images. Therefore, we made the scale between 0 and 1 to be compatible with the methods.

### 2.3. Machine Learning and Deep Learning to Predict Invasive Cancer

In this section, the proposed system is compared to the classic regression techniques and deep learning (DL), with these techniques explained in detail.

### 2.4. Machine Learning Classification Methods for Predicting Invasive Cancer

Classification in ML and statistics is a supervised learning method in which program learns from the given data and then uses it to classify new observations. The dataset is only allowed to be biclass or multiclass [31]. Speech recognition, document classification, biometric identification, handwriting recognition, and so forth are only a few significant examples of classification problems. The proposed system uses the following machine learning (ML) classifiers:

1. Logistic regression
2. *K*-nearest neighbor
3. Support vector machines

#### 2.4.1. Logistic Regression (LR)

Logistic regression is an estimation applied to forecast a binary outcome like either something happens or not. This may be shown as “Yes/No,” “Pass/Fail,” “Alive/Dead,” and so forth. If we consider IDC (+) as 1 and IDC (−) as 0, then the output will be a categorical 0 or 1, which could be defined as

(1) $$\begin{array}{c} P\left(Y=1|X\right)\\ \text{or }P\left(Y=0|X\right). \end{array}$$

This estimates the likelihood of dependent variable *Y*, given independent variable *X*. The decision boundary of logistic regression can be linear or nonlinear, with an increase in the polynomial order resulting in a complex system. The cost function cannot be an *R*-squared function due to its nonconvex structure. Owing to the nature of the cost function in logistic regression (which includes Bernoulli distribution), the dependent variable also follows the same distribution, with this shown in Figure 2.

#### 2.4.2. *K*-Nearest Neighbour (K-NN)

*K*-nearest neighbor (*k*-NN) is an algorithm for pattern recognition which applies training datasets to explore the closest relatives to *k* in future examples. The theory for the nearest-neighbor algorithm is used to define several training samples adjoining to the new point and to use them to forecast the label.

The sample number may be a constant defined by the user, *k*-nearest neighbor (*k*-NN) learning, or may vary according to the local point density. The distance may be any metric measure: standard Euclidean distance is generally a common choice. The nearest neighbor is also available for a large number of datasets due to its simple structure, which can achieve better results for complex boundaries. In Figure 3, the larger values of *K* seem to have a smoother boundary with lower variances.

Euclidean distance is given by

(2) $$\begin{array}{c} d\left(x,y\right)=\sqrt{\sum_{i=1}^{d}{\left(x_{i}-y_{i}\right)}^{2}}, \end{array}$$

for the vector **x** = (*x*_1_,…, *x*_*d*_) has *d* scalar components.

#### 2.4.3. Support Vector Machines (SVM)

It is effective in high-dimensional spaces. In an *n*-dimensional space, each data item is plotted as a point by this algorithm, where *n* denotes the feature number and each feature value indicates a unique coordinate value. It is then possible to carry out classification after getting the hyperplane that best differentiates the two classes, as shown in Figure 4.

### 2.5. Metrics

For the evaluation of machine learning classification models, accuracy is one metric. Accuracy is specified as the percentage of correct predictions for a model. Usually, accuracy is calculated with the following:

(3) $$\begin{array}{c} \text{accuracy}=\frac{\text{number of correct predictions}}{\text{total number of predictions}}. \end{array}$$

Accuracy can also be evaluated as positive and negative for binary classification as follows:

(4) $$\begin{array}{c} \text{accuracy}=\frac{\text{TP}+\text{TN}}{\text{TP}+\text{TN}+\text{FP}+\text{FN}}, \end{array}$$

where TP is used to represent True Positives, TN is used to represent True Negatives, FP is used to represent False Positives, and FN is used to represent False Negatives.

The true positives number divided by the true positives number plus the false positives number is known as precision as shown below:

(5) $$\begin{array}{c} \text{precision}=\frac{\text{TP}}{\text{TP}+\text{FP}}. \end{array}$$

### 2.6. Deep Learning

Deep neural networks usually have several hidden layers in between input layer and output layer. These networks are used to retrieve features from images, unlike traditional ML algorithms which use hand-engineering features for breast cancer detection [32]. A new type of deep learning (DL) is machine learning neural networks (ML-NNs), with ML-NN structures mostly requiring a training stage to find optimum weights. The most frequently used learning rule is the backpropagation algorithm in which weights are updated systematically for every pass depending upon the error rate obtained from the production layer with the gradient and chain rule.

### 2.7. Convolutional Neural Networks (CNNs)

CNNs are applied to explore patterns in an image. This is done by convoluting over an image and looking for patterns [27]. The network can detect lines and corners in the few front layers of CNNs. Via our neural net, however, we can then transfer these patterns down and begin to identify more complex characteristics as we get deeper. This property ensures that CNNs are very effective at detecting objects in images [26]. The proposed system uses CNNs to detect breast cancer from breast tissue images.

The architecture of a CNN has 3 main layers, the convolutional layer, pooling layer, and fully connected layer, as shown in Figure 5. The first layer calculates the output of neurons which are linked with local regions. Each one is calculated by a dot product of weights and the region. For image inputs, typical filters are small in area such as 3 × 3, 5 × 5, or 8 × 8. These filters scan the image by a sliding window on the image, while learning the recurrent patterns which arise in any area of the image. The interval between filters is known as the stride. The convolution is extended to overlapping windows if the stride hyperparameter is smaller than the filter dimension. A detailed visual explanation of neural networks (NNs) is shown in Figure 6.

### 2.8. Pooling Layer

Convolutional layers bring out the features of images with precise positions. If the positions change, even a small amount for any reason, the feature maps will be different. To overcome this problem, the downsampling process must be done at the output of every convolutional layer [18]. With convolutional layers, downsampling can be done by changing the convolution's phase across the image. A more acceptable and common method is to use a pooling layer [33]. Using this process, outputs will be more accurate.

### 2.9. Dataset Augmentation Technique

Data augmentation is an effective and widely used tool to avoid the overfitting problem by creating additional data [34]. More complex systems using deep neural network have low bias but generate high variance. It means that these systems overfit the training data and will demonstrate bad performance on test data or on data that had not seen before. It would result in greater errors in prediction [19]. Therefore, the increased diversity from data augmentation decreases the model's variance by improving it at generalizing. The proposed system uses Gaussian Mixture Models (GMMs) for modeling and classification [35].

## 3. Results and Discussion

We have used scikit-learn machine learning framework for implementation in Python. Scikit-learn is most popular among data scientists. Also, there are other prerequisites to run scikit-learn functions such as pandas, NumPy, matplotlib, and seaborn frameworks which have been used to implement the proposed system.

### 3.1. Predicting Invasive Cancer Using Machine Learning Classifiers

Table 1 presents the accuracies of machine learning (ML) classifiers. The highest level of accuracy is found in SVMs when compared to logistic regression (LR) and *k*-NN, as shown in Figure 7.

### 3.2. Predicting Invasive Cancer Using CNN Model 1

CNN Model 1 has two convolution layers with 32 and 64 kernels, which are checked with a dropout regularization of 25% to cancel overfitting. The image is then vectorized with a flattened layer for the next dense layer. The rectified linear unit (ReLu) is an activation function that is used in all layers with the exception of the output layer, for which the Softmax activation function is used [1].

This model has been trained with 12 epochs and the batch size is 128. The training loss is 0.69, while the validation is 0.68. Little difference is found between model's performances in the training set and the validation set [30].  Table 2 shows the configuration summary of Model 1 with the metrics results presented in Figure 8. It has 59% accuracy, which is less than standard machine learning (ML) classifiers, as shown in Table 3. The loss learning curve is shown in Figure 9.

### 3.3. Predicting Invasive Cancer Using CNN Model 2

To increase the number of features, convolution layers are tripled here [36]. The accuracy of the proposed system is thus increased to 0.76 as shown in Table 4, an improvement on Model 1.  Table 5 shows the configuration summary of Model 2. The confusion matrix and the loss learning curve are shown in Figures 10 and 11, respectively. However, as shown in Figure 11, the validation score is consistently less than the training score, with the suspicion that this model suffers from bias [19].

### 3.4. Predicting Invasive Cancer Using CNN Model 3

CNN Model 3 is deeper than Models 1 and 2, with a five-layer CNN used to detect breast cancer [37]. This architecture gives the best result with 87% accuracy as shown in Table 6: it also provides a similar distribution of predicted labels to that of actual labels (50/50).  Table 7 shows the configuration summary of Model 3. The confusion matrix and the loss learning curve are shown in Figures 12 and 13, respectively.

## 4. Conclusions

Automating the detection of breast cancer to enhance the care of patients is a challenging task. The current study proposes a CNN approach that analyzes the IDC tissue regions in WSIs for the automatic detection of this cancer. Three different CNN architectures have been described in this paper with a proper comparison. The proposed system using CNN Model 3 achieves 87% accuracy. Although Model 3 is deeper than Models 1 and 2, the five-layer CNN in Model 3 is best suited for this task. All architectures were guided by a big dataset of about 275,000, 50 × 50-pixel RGB image patches. When we compared the proposed model with the machine learning (ML) algorithm, the proposed model improved accuracy by 8% over the result of the algorithm. The proposed model was found to successfully obtain correct results that might decrease human mistakes in the diagnosis process and reduce the cost of cancer diagnosis. The main limitation of this study is to use the secondary database like Kaggle, and future study should be done based on primary data for more accuracy of the results related to breast cancer identification.

## Figures and Tables

**Figure 1:** Tissue examples of IDC (+) and IDC (−). (a) IDC (+) tissue and (b) IDC (−) tissue.

**Figure 2:** Linear regression (a) and logistic regression (b).

**Figure 3:** *K* = 1 (a) and *K* = 20 (b) for *k*-nearest neighbour boundaries.

**Figure 4:** SVM formula.

**Figure 5:** Typical CNN architecture for automatic detection of IDC breast cancer.

**Figure 6:** Detailed process of a neural network (NN).

**Figure 7:** Algorithm comparison on accuracy.

**Figure 8:** The confusion matrix of CNN Model 1.

**Figure 9:** The loss learning curve for CNN Model 1.

**Figure 10:** The confusion matrix of CNN Model 2.

**Figure 11:** The loss learning curve for Model 2.

**Figure 12:** Confusion matrix of CNN Model 3.

**Figure 13:** Loss learning curve for Model 3.

**Table 1:** Standard machine learning classifiers.

Classifier	Accuracy
LR	0.7180
KNN	0.7126
SVM	0.7856

**Table 2:** The summary table of CNN Model 1.

Layer	Type	Output shape	Param.
conv2d_2	Conv2D	None, 48, 48, 32	896
conv2d_1	Conv2D	None, 46, 46, 64	18496
max_pooling2d	MaxPooling2D	None, 23, 23, 64	0
Dropout	Dropout	None, 23, 23, 64	0
Flatten	Flatten	None, 33856	0
Dense	Dense	None, 128	4333696
dropout_1	Dropout	None, 128	0
dense_1	Dense	None, 2	258
Total params: 4,353,346			
Trainable params: 4,353,346			
Nontrainable params: 0			

**Table 3:** The metric results of CNN Model 1.

	Precision	Recall	F1-score	Support
IDC (−)	0.59	0.80	0.68	596
IDC (+)	0.60	0.36	0.45	514
Accuracy			0.59	1110

**Table 4:** The metric results of CNN Model 2.

	Precision	Recall	F1-score	Support
IDC (−)	0.72	0.91	0.81	596
IDC (+)	0.85	0.60	0.70	514
Accuracy			0.76	1110

**Table 5:** The summary table of CNN Model 2.

Layer	Type	Output shape	Param.
conv2d_2	Conv2D	None, 50, 50, 32	896
conv2d_3	Conv2D	None, 50, 50, 32	9248
max_pooling2d_1	MaxPooling2	None, 25, 25, 32	0
batch_normalization	BatchNo	None, 25, 25, 32	128
dropout_2	Dropout	None, 25, 25, 32	0
conv2d_4	Conv2D	None, 25, 25, 64	18496
conv2d_5	Conv2D	None, 25, 25, 64	36928
max_pooling2d_2	MaxPooling2	None, 12, 12, 64	0
batch_normalization_1	BatchNo	None, 12, 12, 64	256
dropout_3	Dropout	None, 12, 12, 64	0
conv2d_6	Conv2D	None, 12, 12, 86	49622
conv2d_7	Conv2D	None, 12, 12, 86	66650
max_pooling2d_3	MaxPooling2	None, 6, 6, 86	0
batch_normalization_2	Batch	None, 6, 6, 86	344
dropout_4	Dropout	None, 6, 6, 86	0
flatten_1	Flatten	None, 3096	0
dense_2	Dense	None, 512	1585664
dropout_5	Dropout	None, 512	0
dense_3	Dense	None, 2	1026
Total params.: 1,769,258			
Trainable params.: 1,768,894			
Nontrainable params.: 364			

**Table 6:** CNN Model 3 metric results.

	Precision	Recall	F1-score	Support
IDC (−)	0.82	0.92	0.91	596
IDC (+)	0.86	0.76	0.85	514
Accuracy			0.87	1110

**Table 7:** CNN Model 3 layers.

Layer	Type	Output shape	Param.
conv2d_20	Conv2D	None, 46, 46, 32	2432
max_pooling2d_10	MaxPooling	None, 15, 15, 32	0
conv2d_21	Conv2D	None, 11, 11, 32	25632
max_pooling2d_11	MaxPooling	None, 3, 3, 32	0
dropout_14	Dropout	None, 3, 3, 32	0
flatten_4	Flatten	None, 288	0
dense_8	Dense	None, 64	18496
dropout_15	Dropout	None, 64	0
dense_9	Dense	None, 2	130
Total params.: 46,690			
Trainable params.: 46,690			
Nontrainable params.: 0			

## Data Availability

Datasets analyzed in this study are publicly available. These data can be found at http://www.andrewjanowczyk.com/use-case-6-invasive-ductal-carcinoma-idc-segmentation/.
